The article "Prosthetic valve endocarditis by Trichosporon mucoides: A case report and review of literature" was published in 2020. Journal: Medicine (Baltimore).

# Prosthetic valve endocarditis by *Trichosporon mucoides*: A case report and review of literature

**DOI:** 10.1097/MD.0000000000022584

**Published:** 2020-10-09

**Authors:** Tae Hoon Oh, Sung Un Shin, Soo Sung Kim, Seong Eun Kim, Uh Jin Kim, Seung-Ji Kang, Hee-Chang Jang, Sook In Jung, Jong-Hee Shin, Kyung-Hwa Park

**Affiliations:** a Department of Infectious Diseases, Chonnam National University Hospital; b Department of Infectious Diseases; c Department of Laboratory Medicine, Chonnam National University Medical School, Gwangju, South Korea.

**Keywords:** infective endocarditis, prosthetic valve, *Trichosporon mucoides*

## Abstract

**Nationale:**

*Trichosporon* species are widely distributed in nature and are emerging opportunistic human pathogens. *Trichosporon* infections are associated with superficial cutaneous involvement in immunocompetent individuals to severe systemic disease in immunocompromised patients. Until now, there is no report in infective endocarditis by *Trichosporon mucoides* confirmed by molecular diagnostics

**Patient concerns:**

A 66-year-old man presented with a fever that had occurred for a period of 6 months. He had undergone aortic valve replacement 10 years prior. Transthoracic echocardiography showed vegetations on the prosthetic aortic valve and native mitral valve. *T mucoides* was detected in the cultures of blood and vegetations.

**Diagnosis:**

DNA sequencing using D/D2 region of rRNA and internal transcribed spacer were performed.

**Interventions:**

Infections were successfully controlled with valve replacement and voriconazole plus liposomal amphotericin B therapy.

**Outcomes:**

There has been no sign of recurrence for 18-months after treatment completion.

**Lessons:**

This is the first reported case of infective endocarditis due to *T mucoides*. Clinicians should consider *Trichosporon* species as causative agents of endocarditis in patients who have undergone cardiac surgery.

## 1 Introduction

The genus *Trichosporon* is phenotypically characterized by the development of hyaline, septate hyphae that fragment into oval or rectangular arthroconidia.^[1]^*Trichosporon* species are soil inhabitants, as well as members of the normal flora of the human mouth, gastrointestinal tract, respiratory tract, vagina, skin, and urinary tract.^[2]^ Clinical isolates primarily cause the superficial hair infection, and rarely cause the systemic disease referred to as trichosporonosis.^[3]^ The former *Trichosporon beigelii* (synonym, *Trichosporon cutaneum*), the major pathogen of the genus, refers to 6 species of medical importance in the new nomenclature (*Trichosporon asahii*, *Trichosporon asteroides*, *T cutaneum*, *Trichosporon inkin*, *Trichosporon mucoides*, and *Trichosporon ovoides*) established in 1994.^[4]^ Following recent molecular studies, the genus has undergone major revision and 50 species of *Trichosporon* have been described from different regions of the globe, including 17 with clinical relevance.^[1]^

*T asahii, T asteroides*, and *T mucoides* cause deep invasive infection in the immunocompromised host; *T cutaneum* causes superficial skin infection; *T ovoides* causes superficial infection of the scalp hair; and *T inkin* causes superficial infection of the pubic hair.^[1]^ Invasive infections by *T mucoides* are rare in immunocompetent hosts.^[5–7]^

Here, we describe the first patient with infective endocarditis caused by *T mucoides* and discuss previous reports in which patients were diagnosed with endocarditis due to *Trichosporon* species.

The article "Prosthetic valve endocarditis by Trichosporon mucoides: A case report and review of literature" was published in 2020. Journal: Medicine (Baltimore).

## 2 Case report

In August 2018, a 66-year-old man visited the outpatient clinic for febrile sensations and chills that had been present for 6 months; he also complained of myalgia and dyspnea. The patient had undergone aortic valve replacement and central annuloplasty 10 years prior, due to severe aortic valve stenosis and moderate mitral valve regurgitation. On admission, he had a blood pressure of 100/60 mm Hg, pulse rate of 54 beats/min, respiratory rate of 18 breaths/min, and body temperature of 36.7°C. Physical examination revealed conjunctival hemorrhage in the left eye and petechial eruption on both lower extremities. Laboratory examinations revealed a white blood cell count of 4700/mm^3^ (44.6% neutrophils and 1.1% eosinophils), a hemoglobin level of 13.0 g/dL, and a platelet count of 96,000/mm^3^. Measurement of inflammatory markers showed a C-reactive protein level of 1.55 mg/dL, erythrocyte sedimentation rate of 40 mm/h, and a procalcitonin level of 0.273 ng/mL. Liver function tests showed an alkaline phosphatase level of 102 U/L, aspartate aminotransferase level of 41 U/L, alanine aminotransferase level of 18 U/L, lactate dehydrogenase level of 687 U/L, total bilirubin level of 0.78 mg/dL, and serum albumin level of 3.5 mg/dL. Renal function tests showed a blood urea nitrogen level of 16.5 mg/dL and a serum creatinine level of 1.68 mg/dL. The serum coagulation profiles showed activated partial thromboplastin and prothrombin times of 81.6 and 37.6 seconds, respectively. Transthoracic echocardiography was performed to evaluate infective endocarditis; this examination revealed a mobile mass-like lesion (0.92 × 1.57 cm) at the prosthetic aortic valve and a hypermobile mass-like lesion (0.96 × 0.67 cm) at the mitral valve. Thus, the patient was treated with injections of ceftriaxone and gentamycin. On day 3 of hospitalization, yeast-forming fungi were detected in blood culture; therefore, fluconazole was administered. The yeast-forming fungi were analyzed by sequencing of the internal transcribed spacer (ITS) (including the 5.8S rRNA gene) and D1/D2 regions of the 26S ribosomal DNA. rRNA genes were amplified using the primers pITS-F (5′-GTCGTAACAAGGTTAACCTGCGG-3′) and pITS-R (5′-TCCTCCGCTTATTGATATGC-3′) and NL1 (5′-GCATATCAATAAGCGGAGGAAAAG-3′) and NL4 (5′-GGTCCGTGTTTCAAGACGG-3′),^[8]^ respectively. BLAST search results indicated a 100% match (450/450 bp for ITS, 533/533 bp for D1/D2) with *T mucoides* (GenBank accession nos. KY107341 and KY103030). Commercial matrix-assisted laser desorption/ionization-time of flight mass spectrometry (MALDI-TOF MS) systems, the VITEK MS (bioMérieux, Marcy l’Etoile, France) with Knowledge Base version 3.0, and the MALDI-TOF Biotyper (Bruker Daltonics, Billerica, MA) identified the isolate as *T mucoides*. In vitro studies of susceptibility to amphotericin B, fluconazole, voriconazole, caspofungin, and micafungin were performed by the Clinical and Laboratory Standards Institute document M27-A3 broth microdilution method.^[9]^ The minimal inhibitory concentrations were as follows: amphotericin B, 1 mg/mL; fluconazole, 16 mg/mL; voriconazole, 0.25 μg/mL; caspofungin, >8 μg/mL; and micafungin, >8 μg/mL. On day 7 after admission, the patient's regimen was changed to intravenous voriconazole plus liposomal amphotericin B, due to continuous fever and new conjunctival hemorrhage.

The article "Prosthetic valve endocarditis by Trichosporon mucoides: A case report and review of literature" was published in 2020. Journal: Medicine (Baltimore).

On day 11 of hospitalization, repeat aortic valve replacement, mitral commissurotomy, and removal of the prosthetic ring and pannus were performed. The same fungus (*T mucoides*) was grown from pus from abscesses around the ring. Histopathology of the anterior petechial skin lesions on both lower extremities on day 4 showed mild dermal perivascular chronic inflammation with red cell extravasation, indicative of vasculitis. From suspected onychomycosis on the left big toe on day 5 after admission, a potassium hydroxide preparation was positive, but no causative fungus was isolated.

Liposomal amphotericin B treatment (3 mg/kg) was maintained for 22 days and voriconazole monotherapy was maintained for 3 months. More than 1.5 year after the end of treatment, the patient has shown no evidence of relapse.

## 3 Discussion

Invasive infection due to *Trichosporon* species is rare in immunocompetent hosts, but more common in immunocompromised hosts and shows unfavorable outcome. The optimal therapy for patients with invasive trichosporonosis, such as endocarditis, is unknown. There have been reports of endocarditis caused by *T asahii, T inkin,* and former *T beigelii* (*T cutaneum*), although the *Trichosporon* species were not clearly identified previously.^[10–24]^ Some mycologists continue to designate *T beigelii* as the etiologic agent responsible for clinical disease caused by the Trichosporon yeasts because differentiating between species can be problematic. Here, we have described a first case of successfully treated prosthetic valve endocarditis caused by *T mucoides* in the immunocompetent patient. We also reviewed prior reports of infective endocarditis caused by *Trichosporon* species (Table 1). In the 12 patients who developed prosthetic valve endocarditis among 16 cases (Table 1), clinical symptoms occurred 2 weeks to 10 years after cardiac valve surgery; 1 patient developed endocarditis related to a pacemaker lead, while 3 patients developed native valve endocarditis. The risk factors for *Trichosporon* endocarditis are heart valve surgery, medical device placement in the heart, and intravenous drug use.

The article "Prosthetic valve endocarditis by Trichosporon mucoides: A case report and review of literature" was published in 2020. Journal: Medicine (Baltimore).

**Table 1:** Summary of cases of *Trichosporon* species endocarditis (including the present case).

In literature of *Trichosporon* species endocarditis, species identification was mostly dependent on direct examination of mycelia from specimens. For our patient, the VITEK 2 Yeast identification card system, MALDI-TOF MS, and DNA sequencing were performed and yielded consistent results. However, the VITEK 2 system may be unreliable for the identification of *Trichosporon* species other than *T asahii*^[25]^; therefore, MALDI-TOF may enable rapid identification of fungal species, as an alternative to polymerase chain reaction-based molecular methods.^[26]^

The prognosis is generally poor in patients with infective endocarditis caused by *Trichosporon* species, with a 56% (9/16) mortality rate; 3 patients died before diagnosis (Table 1). Embolic complications were observed in 75% (12/16) of patients and recurrent infection was common. In patients with fungal endocarditis, valve replacement is necessary; however, optimal therapy for patients with invasive trichosporonosis is unknown. The levels of biofilm formation by *Trichosporon* species were greater than those of *Candida*.^[27]^ However, echinocandins, which have a robust anti-*Candida* biofilm effect, are inadequate for *Trichosporon* endocarditis because of intrinsic resistance, as observed in our patient.^[26]^ We applied liposomal amphotericin B plus voriconazole for 3 weeks, followed by voriconazole monotherapy for 3 months with surgery. *T mucoides* is more resistant to fluconazole in vitro, compared to other species.^[28]^ Voriconazole showed the strongest in vitro activity against all *Trichosporon* species.^[29]^ In a study of 55 patients with hematological disease who developed disseminated trichosporonosis and were treated with amphotericin B, only 24% showed a clinical response.^[30]^ Amphotericin B treatment without azoles did not result in favorable outcomes for patients with endocarditis in our literature review (Table 1).

The article "Prosthetic valve endocarditis by Trichosporon mucoides: A case report and review of literature" was published in 2020. Journal: Medicine (Baltimore).

## 4 Conclusions

We reported the first case of patient with infective endocarditis due to *T mucoides*. Clinicians should consider *Trichosporon* species as causative agents of endocarditis in immunocompetent patients who have undergone cardiac surgery. The combination of voriconazole plus amphotericin B may be effective for the treatment of *Trichosporon* endocarditis.

## Author contributions

**Conceptualization:** Kyung-Hwa Park.

**Data curation:** Tae Hoon Oh.

**Investigation:** Kyung-Hwa Park, Tae Hoon Oh, Sung Un Shin, Soo Sung Kim, Seong Eun Kim, Uh Jin Kim, Seung-Ji Kang, Hee-Chang Jang, Sook In Jung, Jong-Hee Shin.

**Supervision:** Kyung-Hwa Park, Sook In Jung, Jong-Hee Shin.

**Writing – original draft:** Tae Hoon Oh.

**Writing – review & editing:** Kyung-Hwa Park, Sook In Jung.

## Abbreviations

Abbreviations: ITS = internal transcribed spacer, MALDI-TOF = matrix-assisted laser desorption/ionization-time of flight mass spectrometry.
